The article "The Healing of Oxidative Injuries with Trehalose in UVB-Irradiated Rabbit Corneas" was retracted in 2020. Reasons: duplicated images; unreliable data; concerns about the images.

# The Healing of Oxidative Injuries with Trehalose in UVB-Irradiated Rabbit Corneas

**DOI:** 10.1155/2019/1857086

**Published:** 2019-09-19

**Authors:** Cestmir Cejka, Jan Kossl, Barbora Hermankova, Vladimir Holan, Sarka Kubinova, Céline Olmiere, Jitka Cejkova

**Affiliations:** ^1^Institute of Experimental Medicine of the Czech Academy of Sciences, Vídenska 1083, 14220 Prague 4, Czech Republic; ^2^Faculty of Natural Science, Charles University, Vinicna 7, 12843 Prague 2, Czech Republic; ^3^Laboratoires Thea (Thea-Pharma), 12 Rue Louis-Bleriot, 63000 Clermont-Ferrand, France

## Abstract

Our previous research revealed that trehalose, a nonreducing disaccharide of glucose and an important stress responsive factor, proved to have anti-inflammatory, antiapoptotic, and particularly antioxidant properties in UVB-irradiated corneas. Trehalose reduced oxidative stress in corneas induced by UVB irradiation, by means of a decrease in the antioxidant/prooxidant imbalance in the corneal epithelium. In this study, we demonstrate that trehalose of 3% or 6% concentration in eye drops directly decreases oxidative stress in UVB-irradiated corneas, by removing the excessive amount of reactive oxygen species (ROS). Trehalose drops applied on corneas during UVB irradiation once daily for four days resulted in a reduction or even absence of the oxidative stress, DNA damage, and peroxynitrite formation (detected by nitrotyrosine residues), seen in buffer-treated corneas. Furthermore, trehalose treatment applied curatively after repeated irradiation for the subsequent fourteen days led to the renewal of corneal transparency and significant suppression or even absence of neovascularization. This was in contrast to buffer-treated irradiated corneas, where the intracorneal inflammation was developed and the untransparent corneas were vascularized. In conclusion, the treatment of UVB-irradiated corneas with trehalose eye drops removed the excessive amount of ROS in the corneal epithelium, leading to the suppression of oxidative stress and favorable corneal healing. The 6% trehalose showed a higher intensive antioxidant effect.

## 1. Introduction

UVB radiation (ultraviolet B, 280-320 nm ray wavelength) induces ROS generation, which in turn causes cellular damage, intracorneal inflammation, changes in corneal hydration, thinning of the corneal epithelium, and an increased appearance of apoptosis [1, 2]. In the UVB-irradiated corneas, the antioxidant/prooxidant imbalance and oxidative stress appear [1, 3–5]. ROS which are insufficiently cleaved, contribute to the increased activities of proteolytic enzymes and the profound induction of proinflammatory cytokines [6–9], resulting in the development of excessive intracorneal inflammation, neovascularization, and changes in corneal optics. ROS play an important role in cellular homeostasis, whereas pathologically high concentrations are associated with cell death, various pathological states, and aging. In seriously injured corneas, ROS can activate the transcription factor NF-*κ*B, which then translocates to the nucleus to induce the expression of proinflammatory cytokines [10].

The article "The Healing of Oxidative Injuries with Trehalose in UVB-Irradiated Rabbit Corneas" was retracted in 2020. Reasons: duplicated images; unreliable data; concerns about the images.

Our previous research showed that trehalose, a disaccharide of glucose, reduced the UVB-induced oxidative stress through the decrease in the antioxidant/prooxidant imbalance in the irradiated corneal epithelium, leading to the decreased overexpression of proinflammatory cytokines, matrix metalloproteinases, and heat shock protein 70. In addition, trehalose decreased cell apoptosis and suppressed corneal inflammation and neovascularization evoked by UVB rays [11–13]. The favorable effect on corneal epithelial cells by trehalose was also described by Aragona et al. [14] and by Hill-Bator et al. [15]. Chen et al. [16] determined the therapeutic effect of trehalose in dry eye disease. Takeuchi et al. [17, 18] investigated the fact that trehalose inhibited vascular endothelial growth factor (VEGF) and the proliferation of myofibroblasts. These findings suggest that trehalose has the potential for use as a new agent that can control angiogenesis and fibrosis and could also be useful in ocular surgery. Kudo et al. [19] demonstrated the inhibitory effect of trehalose on malignant melanoma cell growth, suggesting trehalose as a potent anticancer agent.

Trehalose is a stress response factor synthetized by many organisms when cells are exposed to various stresses, including dehydration, heat, oxidation, hypoxia, or even anoxia [20]. Trehalose is not synthesized by mammalian cells, but it does however reveal a number of unique properties that indicate its utility in humans [21]. Trehalose is effective in wound healing by protecting cells, especially cell membranes, from oxidative injury and desiccation [11, 12, 15, 16, 22].

In this study, we compared the efficacy of two concentrations of trehalose (3% and 6%) on the healing of UVB-irradiated corneas. The results showed that both concentrations of trehalose used during UVB irradiation decreased oxidative stress in irradiated corneas by removing an excessive amount of ROS. The 3% trehalose concentration reduced oxidative stress and DNA damage, whereas after the treatment with 6% trehalose, oxidative stress and DNA damage were prevented. Trehalose drops applied on corneas after UVB irradiation for two weeks healed the corneal oxidative injuries without untransparent scar formation. The higher trehalose concentration was more effective.

The article "The Healing of Oxidative Injuries with Trehalose in UVB-Irradiated Rabbit Corneas" was retracted in 2020. Reasons: duplicated images; unreliable data; concerns about the images.

## 2. Materials and Methods

### 2.1. Trehalose Eye Drops

Trehalose eye drops of 3% and 6% concentration and buffer eye drops were kindly supplied from Laboratoires Thea, Clermont-Ferrand, France.

### 2.2. Experimental Animals and UVB Irradiation

The investigation was conducted according to the ARVO Statement on the Use of Animals in Ophthalmic and Vision Research. Adult female New Zealand white rabbits (2.5-3.0 kg) were divided into two groups for the experiments, with six rabbits for 3% and six rabbits for 6% of trehalose concentration in each group and six rabbits for a control group with buffer drops. All the experiments were repeated twice. The rabbits were anesthetized by an intramuscular injection of Rometar (Xylazinum hydrochloricum, Spofa, Prague, CR, 2%, 0.2 ml/kg body weight) and Narkamon (Ketaminum hydrochloricum, Spofa, 5%, 1 ml/kg body weight). The open eyes of the anesthetized rabbits were irradiated (right eyes of each rabbit) with a UVB lamp (Bioblock Scientific, Illkirch Cedex, France; 312 nm wavelength, 6 W), with a dose of 0.5 J/cm^2^ per day for four days. The irradiation took place from a distance of 0.06 m for 5 min. A UV lamp stand was used with an exact determined distance between the lamp and the eye of the animal. The plane of the lamp was parallel to the tangential plane of the eye (perpendicular to the optical axis of the eye). The intensity and total dose of irradiation were regularly measured with a UVB sensor connected to a radiometer (both instruments manufactured by Cole-Parmer Inc., Vernon Hills, Illinois, USA). Although the source of UVB that was used emits only UVB rays peaking at 312 nm (according to the irradiation spectrum given by the manufacturer), a UVC sensor (Cole-Parmer Inc.) was used to check for the potential emission of UVC light. During irradiation, the eyes of the anesthetized animals were held open. Only the corneas were irradiated, and the rest of the ocular surface was protected with a sterile gauze (slightly soaked with Aqua Pro injection for softening) with the central hole of the same diameter as the rabbit cornea.

In the first group of experiments, the animals were treated during the four days of daily irradiation with 3% or 6% trehalose or with buffered saline, with three drops put in each eye six times daily. After the irradiation procedures (day 4 of repeated irradiation), the animals were sacrificed under i.v. injection of thiopental anesthesia (thiopental, Spofa, 30 mg/kg following premedication with i.m. Rometar/Narkamon) and the excised corneas were employed for the measurement of ROS and for the immunohistochemical examinations. In the second group of experiments, the animals were repeatedly irradiated with UVB rays for four days (as described above); however, the treatment with 3% or 6% trehalose or buffered saline followed the irradiation procedures and continued for fourteen days, with three drops put in each eye, four times daily (Figure 1). After the treatment had finished, the animals were sacrificed and the corneas microscopically and biochemically examined. Normal corneas from untreated animals served as controls. During the whole experiment, the eyes were photographically documented and the central corneal thickness was measured with an ultrasonic pachymeter.

The article "The Healing of Oxidative Injuries with Trehalose in UVB-Irradiated Rabbit Corneas" was retracted in 2020. Reasons: duplicated images; unreliable data; concerns about the images.

### 2.3. Measurement of Reactive Oxygen Species (ROS)

On the fourth day of UVB irradiation of rabbit corneas, the animals were sacrificed and the eyeballs were enucleated, the anterior eye segments were immediately frozen in light petroleum chilled with an acetone-dry ice mixture, and sections were cut on a cryostat and transferred onto glass slides. The unfixed cryostat sections were incubated with 5 *μ*M dihydroethidium (DHE, Sigma, Saint Louis, MO, USA) for 15 min at 37°C. Sections were examined with a Leitz Orthoplan light microscope equipped with a Leica DC 500 digital camera, and the intensity of staining was measured using the Fiji ImageJ Program [23].

### 2.4. The Determination of the Corneal Thickness

Changes of corneal optical properties after the injury and during healing were evaluated by measuring the central corneal thickness (taken as an index of corneal hydration) (see [24] in detail). Briefly, the central corneal thickness was measured in anesthetized animals using an ultrasonic pachymeter SP-100 (Tomey Corporation, Nagoya, Japan) in the corneal center. The corneal thickness was measured in the same corneas before irradiation (corneas of healthy eyes) and in individual time intervals in all experimental groups. Each cornea was measured four times, and the mean value and SD of the thickness (in *μ*m) were computed.

### 2.5. Evaluation of Corneal Neovascularization and Transparency

For evaluation of corneal neovascularization, the number of vessels was counted in each of the 60° sectors of the corneal surface. The mean value and standard deviation were counted from five measurements. This procedure was applied for every eye from a matching group of eyes.

### 2.6. Immunohistochemistry and Immunofluorescence

After sacrificing the animals, the eyes were enucleated and the anterior eye segment was dissected and quenched in light petroleum, chilled with an acetone-dry ice mixture. Sections were cut on a cryostat and transferred onto glass slides. Subsequently, the cryostat sections were fixed in acetone at 4°C for 5 min. For the immunohistochemical detection of 8-hydroxyguanosine (8-OHdG), interleukin-1*β* (IL-1*β*), vascular endothelial growth factor (VEGF), inducible nitric oxide synthase (iNOS), or cytokeratins K3 and K12 (K3/12), the following primary monoclonal antibodies were used: anti-8-OHdG (Abcam, http://www.abcam.com), anti-IL-1*β* (Thermo Fisher Scientific, https://www.thermofisher.com/cz/en/home/life-science/antibodies.html), anti-iNOS (BD Biosciences, San Jose, CA, USA), anti-K3/12 (Abcam), and anti-VEGF (Abcam). The binding of the primary antibodies was demonstrated using the horseradish peroxidase/3,3′-diaminobenzidine (HRP/DAB) Ultra Vision detection system (Thermo Fisher Scientific) following the instructions of the manufacturer. Individual steps involved the following: hydrogen peroxide block (15 min), ultra V block (5 min), incubation with the primary antibody (60 min), incubation (10 min) with a biotinylated goat anti-mouse IgG secondary antibody (Thermo Fisher Scientific), and peroxidase-labeled streptavidin incubation (10 min). Visualization was performed using a freshly prepared DAB substrate-chromogen solution. Cryostat sections in which the primary antibodies were omitted from the incubation media served as negative controls. Some sections were counterstained with Mayer's hematoxylin. For the detection of nitrotyrosine (NT) by immunofluorescence, the post-fixed cryostat sections (in acetone at 4°C for 5 min) were incubated (60 min) with mouse anti-nitrotyrosine (1 : 100, Abcam), followed by 45 min incubation with Alexa Fluor 488 goat anti-mouse IgG. After the procedure, the samples were immediately examined under the microscope (Leitz).

The article "The Healing of Oxidative Injuries with Trehalose in UVB-Irradiated Rabbit Corneas" was retracted in 2020. Reasons: duplicated images; unreliable data; concerns about the images.

### 2.7. Detection of Gene Expression by Real-Time PCR

The expression of genes for K3, iNOS, IL-1*β*, and VEGF in the control and treated corneas was determined by quantitative real-time polymerase chain reaction (PCR). The corneas were excised using Vannas scissors, transferred into Eppendorf tubes, and immediately frozen. The frozen corneal tissue was then homogenized and added in 500 *μ*l of TRI Reagent (Molecular Research Center, Cincinnati, OH, USA) for the RNA isolation. The RNA isolation and transcription and the PCR parameters were performed as follows. The total RNA was extracted using TRI Reagent according to the manufacturer's instructions. 1 *μ*g of total RNA was treated using deoxyribonuclease I (Promega, Madison, WI, USA) and subsequently used for reverse transcription. The first-strand cDNA was synthesized using random primers (Promega) in a total reaction volume of 25 *μ*l, using M-MLV Reverse Transcriptase (Promega). Quantitative real-time PCR was performed in a StepOnePlus real-time PCR system (Applied Biosystems, Foster City, CA, USA). A relative quantification model with efficiency correction was applied to calculate the expression of the target gene in comparison with GAPDH used as the housekeeping gene. The following primers were used for amplification: GAPDH: 5′-CCCAACGTGTCTGTCGTG (sense) and 5′-CCGACCCAGACGTACAGC (antisense), K3: 5′′-GAACAAGGTCCTGGAGACCA (sense) and 5′-TTGAAGTCCTCCACCAGGTC (antisense), iNOS: 5′-AGGGAGTGTTGTTCCAGGTG (sense) and 5′TCCTCAACCTGCTCCTCACT (antisense), IL-1*β*: 5′-CTGCGGCAGAAAGCAGTT (sense) and 5′-GAAAGTTCTCAGGCCGTCAT (antisense), and VEGF: 5′-CGAGACCTTGGTGGACATCT (sense) and 5′-ATCTGCATGGTGACGTTGAA (antisense). The PCR parameters included denaturation at 95°C for 3 min, then 40 cycles at 95°C for 20 s, annealing at 60°C for 30 s, and elongation at 72°C for 30 s. Fluorescence data were collected at each cycle after an elongation step at 80°C for 5 s and were analyzed using the StepOne Software, version 2.2.2 (Applied Biosystems). Each individual experiment was done in triplicate.

The article "The Healing of Oxidative Injuries with Trehalose in UVB-Irradiated Rabbit Corneas" was retracted in 2020. Reasons: duplicated images; unreliable data; concerns about the images.

### 2.8. Statistical Analysis

Analysis of the data showed normal distribution, and the results are expressed as mean ± SD. Comparisons between the two groups were made by the Student *t*-test, and multiple comparisons were analyzed by ANOVA. A value of *P* < 0.05 was considered statistically significant.

## 3. Results

### 3.1. Graphical Schemes for the Program of Experiments Are Shown in Figure 1.

### 3.2. The Effect of Trehalose Treatment on the ROS Production

Dihydroethidium (DHE) fluorescence staining, as an indicator of ROS production, was detected in the control corneas and irradiated corneas treated with trehalose eye drops (3% or 6%) or buffer drops. The measurement of DHE fluorescence intensity demonstrated that trehalose treatment significantly decreased ROS production in UVB-irradiated corneas, compared to corneas treated with buffer drops (Figures 2(a) and 2(b)). The 6% trehalose reduced ROS production more than the 3% trehalose.

### 3.3. The Effect of Trehalose Treatment on DNA Damage and Nitrotyrosine Staining

Immunohistochemical detection of the 8-hydroxyguanosine (8-OhdG) and nitrotyrosine (NT) was performed in control corneas and corneas treated with trehalose (3% or 6%) or buffer drops after four days of daily UVB irradiation.

The immunohistochemical expression of 8-OhdG and NT was intense in buffer-treated corneas (Figures 3(d) and 3(h)) and reduced in corneas treated with 3% trehalose (Figures 3(b) and 3(f)). No substantial expression of 8-OhdG and NT was visible in corneas treated with 6% trehalose (Figures 3(c) and 3(g)), similarly as in the control intact cornea (Figures 3(a) and 3(e)).

The article "The Healing of Oxidative Injuries with Trehalose in UVB-Irradiated Rabbit Corneas" was retracted in 2020. Reasons: duplicated images; unreliable data; concerns about the images.

### 3.4. The Effect of Trehalose Treatment on Expression of K3/K12, iNOS, IL-1*β*, and VEGF

Immunohistochemical detection and gene expression of K3/K12, IL-1*β*, VEGF of K3, and VEGF were analyzed in UVB-irradiated corneas of rabbits treated with trehalose (3% or 6% concentration) or buffer, for fourteen days after the end of repeated irradiation (daily for 4 days).

UVB-irradiated corneas quickly reepithelialized (expressed by K3/K12 staining) after the treatment with 3% trehalose (Figure 4(b)) and even more after the treatment with 6% trehalose (Figure 4(c)), whereas after the treatment with buffer drops, corneas were almost without the epithelium (Figure 4(d)). Gene expression for cytokeratin K3 was detected in control and trehalose-treated corneas but absent or very low in corneas treated with buffer drops (Figure 4(e)).

The expression of iNOS and IL-1*β* was not detected in control corneas (Figures 5(a) and 5(b)) but was remarkably high in buffer-treated corneas (Figures 5(g) and 5(h)). iNOS and IL-1*β* staining intensity was decreased in corneas treated with 3% trehalose (Figures 5(c) and 5(d)) and nearly absent in corneas treated with 6% trehalose (Figures 5(e) and 5(f)). Gene expression for IL-1*β* (Figure 6(j)) and iNOS (Figure 5(i)) was apparent in buffer-treated corneas, whereas it was very low or absent in trehalose-treated corneas. The expression of VEGF was high in buffer-treated corneas (Figure 6(d)), whereas in corneas treated with 3% trehalose, it was low (Figure 6(b)), and in corneas treated with 6% trehalose (Figure 6(c)), it was absent. Similarly, gene expression of VEGF was the highest in buffer-treated corneas and decreased in corneas treated with 3% trehalose and was nearly absent in corneas treated with 6% trehalose (Figure 6(e)). Corneal neovascularization (the number of vessels per sector) is summarized in Figure 6(f).

### 3.5. Macroscopical Images of UVB-Irradiated Corneas after Trehalose Treatment and the Central Corneal Thickness

Macroscopical images of the eyes were taken after four days of repeated irradiation with UVB rays and simultaneous treatment with 3% and 6% trehalose or buffer during irradiation and after repeated UVB irradiation for four days and subsequent treatment with 3% and 6% trehalose or buffer for fourteen days. Macroscopical images were completed with changes in the central corneal thickness measured with an ultrasonic pachymeter.

In Figure 7(a), macroscopical images of corneas repeatedly irradiated with UVB rays for four days and treated during irradiation with buffer drops lost transparency, and corneas turned white and were vascularized. After the treatment with trehalose, corneas remained transparent and neovascularization was highly suppressed after 3% trehalose or was even absent after 6% trehalose treatment. In Figure 7(b), the central corneal thickness of corneas irradiated for four days (once daily) is summarized. When buffer eye drops were applied during irradiation, the central corneal thickness was gradually increasing. Trehalose treatment during irradiation (more after drops of higher trehalose concentration) decreased the central corneal thickness.

The article "The Healing of Oxidative Injuries with Trehalose in UVB-Irradiated Rabbit Corneas" was retracted in 2020. Reasons: duplicated images; unreliable data; concerns about the images.

In Figure 7(c), following two weeks of treatment of UVB-irradiated corneas (once daily for four days), the untransparent corneas were healed with the restoration of transparency after the treatment with 3% trehalose and corneal neovascularization was highly suppressed, whereas treatment with 6% trehalose prevented the corneal neovascularization. In contrast, after the treatment with buffer drops, corneas healed with untransparent scar tissue and apparent neovascularization.  Figure 7(d) summarizes the central corneal thickness of corneas irradiated with UVB rays for four days (once daily) without any treatment and then treated with buffer or trehalose drops for fourteen days. Trehalose drops significantly decreased the levels of the corneal thickness.

## 4. Discussion

UVB irradiation induces an acute corneal inflammation, photokeratitis, accompanied by ROS generation, an increase in corneal thickness, and a decrease in antioxidants [3, 4]. In this study, the efficacy of lower and higher trehalose concentrations was examined in two experiments of UVB-irradiated corneas (Figure 1). The results show that both concentrations of trehalose revealed potent antioxidative and anti-inflammatory properties. Trehalose directly removed the excessive amount of ROS in irradiated corneas. Trehalose of higher concentration was more effective in these processes. Although the treatment with trehalose of lower concentration suppressed oxidative stress and DNA damage in corneas, the treatment with trehalose of higher concentration prevented these processes. Previous research, confirmed in this study, has shown that irradiation of corneas with UVB rays evokes oxidative stress in corneas [1, 3, 5] (Figure 2). Oxidative stress is involved in a number of human corneal diseases and ocular surface inflammatory diseases, including dry eye disease [25–27]. Oxidative stress is caused by an imbalance between the production of ROS and their removal. Repeated UVB radiation induced an excessive generation of ROS leading to a decrease in antioxidants, whereas prooxidants remained at normal levels or even increased [1, 3, 5]. This antioxidant/prooxidant imbalance, together with the more pronounced production of nitric oxide generated by nitric oxide synthases, led to the formation of cytotoxic nitrogen-related oxidants, such as peroxynitrite, generated by the rapid reaction of nitric oxide with superoxide [6]. Trehalose has shown broad antioxidant properties. Mizunoe et al. [28] described how trehalose protects against oxidative stress by regulating the Keap1-Nrf2 and autophagy pathways. We believe this study is the first to show that trehalose directly reduces the excessive amount of ROS in irradiated corneas (DHE assay, Figure 2). Comparable results were found with the NT expression and DNA damage (shown by the expression of 8-OHdG, Figure 3). ROS, produced either endogenously or exogenously, can attack lipid, protein, and nucleic acid simultaneously in the living cells. In nuclear and mitochondrial DNA, 8-OHdG, an oxidized nucleoside of DNA, is the most sensitive biomarker to determine oxidative DNA damage [29]. According to Tsai et al. [30] among numerous types of oxidative DNA damage, the formation of 8-OHdG presents only a minor fraction of UV-induced DNA damage, but it is a ubiquitous marker of oxidative stress. When trehalose treatment of corneas was started, after the end of repeated corneal irradiation, and the corneal epithelium was damaged or even lost, the reepithelialization of corneas quickly continued, particularly after the application of trehalose of higher concentration (Figure 4). The intracorneal inflammation developed in buffer-treated UVB-irradiated corneas, as shown using the expression of IL-1*β*, was significantly reduced after the trehalose treatment (3% concentration) and absent after the higher trehalose concentration (6%) (Figure 5). Corneas healed with the restoration of transparency. The central corneal thickness (taken as an index of corneal hydration) was decreased after trehalose treatment. Changes of corneal hydration are important markers of corneal healing and transparency [31]. Corneal neovascularization was decreased after the treatment with 3% trehalose and nearly absent after the treatment with 6% trehalose (Figures 6 and 7).

The article "The Healing of Oxidative Injuries with Trehalose in UVB-Irradiated Rabbit Corneas" was retracted in 2020. Reasons: duplicated images; unreliable data; concerns about the images.

## 5. Conclusions

In severe oxidative damage, such as corneal photodamage, following the irradiation of corneas with UVB rays, the trehalose eye drops of higher concentration (6%) showed more effective antioxidant properties than the trehalose of lower concentration (3%). The higher concentration of trehalose significantly suppressed corneal oxidative stress by removing ROS and prevented DNA damage and peroxynitrite formation in irradiated corneas, resulting in rapid healing without corneal scar formation and neovascularization. Trehalose is an important nontoxic drug which effectively protects cells and tissues against oxidative stress.

## Figures and Tables

**Figure 1:** Graphical scheme of the program of experiments with corneal UVB irradiation and experimental groups treated with buffer or trehalose drops is shown.

**Figure 2:** Production of reactive oxygen species (ROS) in the UVB-irradiated corneas (once daily for 4 days) treated with buffer or 3% or 6% trehalose eye drops examined by the dihydroethidium (DHE) assay. The intensity of fluorescence was scaled by integral optical density. (a) Compared to buffer-treated corneas, the oxidative stress in the corneal epithelium was reduced by 3% trehalose and strongly suppressed by 6% trehalose. (b) In the corneal epithelium treated with buffer alone, the intensity of fluorescence was significantly higher compared to that of fluorescence of the control epithelium or corneal epithelium treated with trehalose eye drops. The values with asterisks are significantly different (^∗^*P* < 0.1, ^∗∗^*P* < 0.01) from those of buffer-treated corneas. Buffer: 80.97 ± 14.6; 3% trehalose: 53.95 ± 7.6; 6% trehalose: 36.46 ± 9.8; control 33.54 ± 7.7; *n* = 5/group. Scale bars: 50 *μ*m.

**Figure 3:** Immunohistochemical detection of 8-hydroxyguanosine (8-OhdG) and immunofluorescence of nitrotyrosine (NT) in the UVB-irradiated corneas (daily for 4 days) treated with buffer or 3% or 6% trehalose eye drops. In control corneas, the expression of 8-OhdG (a) and immunofluorescence of NT (e) are practically absent, similarly as after the treatment of UVB-irradiated corneas with drops of 6% trehalose (arrows) (8-OhdG (c), NT (g)). A slightly increased expression of 8-OhdG (arrows) (b) and of NT (f) (arrows) is seen after the treatment with 3% trehalose. The treatment with buffer drops induces the distinct expression (arrows) of 8-OhdG (d) and NT (h) in irradiated corneas. Scale bars: 50 *μ*m.

**Figure 4:** Corneal reepithelialization shown by the expression of K3 and K12 in UVB-irradiated corneas of rabbits treated with trehalose drops (3% or 6%) or buffer drops for fourteen days after the end of repeated UVB irradiation. Sections are counterstained with hematoxylin. The individual pictures show the representative images of anti-K3/12-stained control cornea (a) and cornea treated with 3% trehalose (b) or 6% trehalose (c) drops or with buffer drops (d). After the treatment of eyes with trehalose, the corneas were reepithelialized. In contrast, after the treatment with buffer drops, corneas were reepithelialized with the flat epithelium or remain without the epithelium. Scale bars: 50 *μ*m. The quantification of corneal reepithelialization with investigation of K3 genes by real-time-PCR is shown in (e). Each bar represents the mean ± SD from 6 corneas. The values with asterisks are significantly different (^∗∗∗^*P* < 0.001) from those of buffer-treated corneas.

The article "The Healing of Oxidative Injuries with Trehalose in UVB-Irradiated Rabbit Corneas" was retracted in 2020. Reasons: duplicated images; unreliable data; concerns about the images.

**Figure 5:** The immunohistochemical expressions of iNOS and IL-1*β* in UVB-irradiated corneas of rabbits treated with trehalose (3% or 6% concentration) drops or buffer drops for fourteen days after the end of repeated irradiation. The expressions of iNOS and IL-1*β* are nearly absent in control corneas (a, b) and in the irradiated corneas treated with 6% trehalose (e, f). In corneas treated with 3% trehalose (c, d), slight expressions of iNOS and IL-1*β* are present. In contrast, after the treatment of corneas with buffer drops, iNOS and IL-1*β* are highly expressed in corneas (g, h). Scale bars: 50 *μ*m. The expression of genes for iNOS and IL-1*β* summarized are shown (i, j). The values with asterisks are significantly different (^∗∗^*P* < 0.01, ^∗∗∗^*P* < 0.001) from those of buffer-treated corneas.

**Figure 6:** The immunohistochemical expression of VEGF and corneal neovascularization in UVB-irradiated corneas of rabbits treated with trehalose (3% or 6% concentration) drops or buffer drops for fourteen days after the end of repeated irradiation. The expression of VEGF is absent in control corneas (a) and nearly absent in UVB-irradiated corneas treated with drops of 6% trehalose (c). Slight expression of VEGF is seen in corneas treated with 3% trehalose (arrow) (b). In contrast, after the treatment of UVB-irradiated corneas with buffer drops, VEGF is highly expressed in corneas (arrow) (d). Scale bars: 50 *μ*m. The quantification of VEGF genes by real-time PCR is shown in (e). Each bar represents the mean ± SD from 6 corneas. The values with asterisks are significantly different (^∗^*P* < 0.05, ^∗∗∗^*P* < 0.001) from those of UVB-irradiated buffer-treated corneas. Quantification of corneal neovascularization (number of vessels) is summarized in (f). Trehalose treatment highly suppressed corneal neovascularization. Each bar represents the mean ± SD from 6 corneas. The values with asterisks are significantly different (^∗∗∗^*P* < 0.001) from those of buffer-treated UVB-irradiated corneas.

**Figure 7:** Representative images and central corneal thickness of corneas treated with trehalose or buffer drops during repeated UVB irradiation and images of corneas treated with trehalose or buffer drops for fourteen days after the finished repeated UVB irradiation. (a) In the first group of corneas (corneas treated during irradiation), the best healing effects were obtained with the treatment with 6% trehalose, followed by the treatment with 3% trehalose. In (b), the central corneal thickness of these corneas is summarized. In trehalose-treated irradiated corneas, the values for days two and four are statistically different (^∗^*P* < 0.1, ^∗∗∗^*P* < 0.001) from the values of buffer-treated corneas. (c) In the second group, when corneas were at first irradiated (for 4 days) and then treated with buffer drops or trehalose drops (for 14 days), the best healing results were also obtained with 6% trehalose, followed by 3% trehalose. Corneal neovascularization was highly suppressed and corneal transparency restored. In contrast, after the treatment of UVB-irradiated corneas with buffer drops, corneas healed with untransparent scar tissue and corneal neovascularization appeared (arrow). Comparison with the control eye. (d) The central corneal thickness of corneas irradiated (for 4 days) and then treated with buffer drops or trehalose drops (for 14 days). The central corneal thickness after trehalose treatment on days ten and fourteen was statistically different (^∗∗∗^*P* < 0.001) from the values of buffer-treated corneas. After the treatment with 6% trehalose, the values of the central corneal thickness on day fourteen reached the values before injury.

The article "The Healing of Oxidative Injuries with Trehalose in UVB-Irradiated Rabbit Corneas" was retracted in 2020. Reasons: duplicated images; unreliable data; concerns about the images.

## Data Availability

The data used to support the findings of this study are available from the corresponding author upon request.

## Abbreviations

DHE: Dihydroethidium
ROS: Reactive oxygen species
NT: Nitrotyrosine
K3, K12: Cytokeratins K3, K12
IL-1*β*: Interleukin-1*β*
*Ι*L- 6: Interleukin-6
iNOS: Inducible nitric oxide synthase
VEGF: Vascular endothelial growth factor
8-OHdG: 8-Hydroxyguanosine
SD: Standard deviation.
